# Research on Lane a Compensation Method Based on Multi-Sensor Fusion

**DOI:** 10.3390/s19071584

**Published:** 2019-04-02

**Authors:** Yushan Li, Wenbo Zhang, Xuewu Ji, Chuanxiang Ren, Jian Wu

**Affiliations:** 1 College of Transportation, Shandong University of Science and Technology, Qingdao 266590, China; skd992034@sdust.edu.cn (Y.L.); Zhangwb@sdust.edu.cn (W.Z.); renchx@sdust.edu.cn (C.R.); 2 State Key Laboratory of Automotive Safety and Energy, Tsinghua University, Beijing 100084, China; 3 School of Mechanical and Automotive Engineering, Liaocheng University, Liaocheng 252059, China; wujian@lcu.edu.cn

**Keywords:** sensor fusion, kinematics, lane detection, vision, virtual lane

## Abstract

The curvature of the lane output by the vision sensor caused by shadows, changes in lighting and line breaking jumps over in a period of time, which leads to serious problems for unmanned driving control. It is particularly important to predict or compensate the real lane in real-time during sensor jumps. This paper presents a lane compensation method based on multi-sensor fusion of global positioning system (GPS), inertial measurement unit (IMU) and vision sensors. In order to compensate the lane, the cubic polynomial function of the longitudinal distance is selected as the lane model. In this method, a Kalman filter is used to estimate vehicle velocity and yaw angle by GPS and IMU measurements, and a vehicle kinematics model is established to describe vehicle motion. It uses the geometric relationship between vehicle and relative lane motion at the current moment to solve the coefficient of the lane polynomial at the next moment. The simulation and vehicle test results show that the prediction information can compensate for the failure of the vision sensor, and has good real-time, robustness and accuracy.

## 1. Introduction

In recent years, intelligent driving vehicles have received widespread attention. The reason is that intelligent driving vehicles can play a positive role in the daily traffic environment. The reliability of intelligent driving control system with mature technology is higher than that of drivers with different driving skills. Important functions of intelligent driving, such as lane keeping systems (LKAs) and lane change systems (LCXs) have been widely studied. In order to ensure autonomous vehicles can drive safely on the road, high-precision lane level location is required. Currently, lane-level location can be realized through Lidar, GPS/INS or cameras. However, the cost of Lidar is higher than that of other sensors. When GPS and INS are used for high-precision positioning, the absolute position information is obtained, which must be matched with a high-precision map to obtain the relative road position information. Therefore, high-efficiency and low-cost environmental perception based on vision will become the main direction of future industrialization of intelligent driving vehicles [1].

Lane recognition [2,3] is an important part of lane-level location. At present, the mainstream method is to obtain lane images through vision sensors installed on intelligent vehicles, and then use the edge, color, texture or frequency domain features of lanes to separate lane lines from road areas. According to the different image processing strategies of road conditions, existing methods can generally be divided into model-based methods [4,5,6,7,8] and feature-based methods [9,10,11,12,13]. However, the acquisition of lane information from vision sensors may fail due to complex shadows, missing lane markers, changes in lighting, different lane brightness or vision sensor failures [14]. In these abnormal conditions, the sensor recognition algorithm automatically chooses to exit temporarily. Based on this kind of problem, scholars have put forward two main solutions. One method is to compensate from the level of image processing. A method using a fuzzy system and line segment detector algorithm to overcome various lighting problems has been presented in [15]. References [16,17,18,19,20,21] respectively improve the robustness of lane recognition in different environments from the aspects of clustering, feature extraction and curve fitting. These methods based on image processing can improve the accuracy of lane detection to a certain extent, but this kind of method is limited by the sensor accuracy. Another method is to improve the robustness of vision sensors by using sensor fusion. A positioning system combining global positioning system (GPS), inertial measurement unit (IMU), wheel speed sensor, single front-facing camera and digital map was proposed in [22,23,24,25,26,27,28,29]. This kind of method relies on digital maps and increases the computational burden of the computer. References [30,31] used a kinematics model of the vehicle and the position information of the vehicle in front based on radar or V2X to predict the lane. However, this method places high requirements on knowing the trajectory of the vehicle in front. A vehicle kinematic lateral motion model and road constraints are used to solve sensor failures in [32,33,34,35]. The kinematics model and dynamics model are combined for lane prediction in the high speed range in [36]. Nevertheless, the above method requires high precision of the model, and the accuracy of the model is related to the performance of the system. Therefore, how to realize information compensation under the condition of discontinuous lane signals is still an important technical problem. The importance of lane information stability to vehicle automatic control is verified in [37,38,39,40]. A real-time vision sensor compensation algorithm will ensure that the movement trajectory of the vehicles can remain stable when the positioning signal is lost, and a sufficient system response time can be provide when the lane information continues to fail. Therefore, it can complete driver wake-up and control transfer, and transfer the control of the vehicle to the driver smoothly and safely.

In this paper, a lane prediction system based on sensor fusion for vision sensor failures has been presented. First, a low-cost GPS, IMU and DR are integrated to obtain a high-precision vehicle trajectory. Secondly, in the multi-sensor system, the relative position relation of the vehicle path is used to predict the lane coefficient, and the prediction algorithm is synchronized with the control sample time. Therefore, when the sensor does not fail, the method proposed in this paper can also verify the lane information which is collected by visual sensors under normal circumstances. Finally, the performance of the method is evaluated by a HIL simulation and vehicle tests at a test site. The proposed method can effectively realize the compensation of vision sensors in the state of failure. The method works effectively after 1 s. Even if the vision sensor breakdown occurs on a bend, this time is enough for the driver to take over control.

The rest of this paper is organized as follows: in Section 2, a low-cost GPS and IMU are used to estimate the vehicle state, and the vehicle trajectory is fitted by dead reckoning based on the vehicle kinematics. The lane coefficient is predicted by using the relative position relationship between the vehicle trajectory and the lane in the multi-rate system in Section 3. The simulation and the experimental results are given in Section 4. Finally, Section 5 outlines the conclusions and discusses the limitations of this method and possible future work.

## 2. Sensor Fusion and Lane Modeling

The GPS, IMU fusion algorithm, vehicle kinematics based on a dead reckoning method, and lane polynomial function are described in this part. More accurate yaw angle and longitudinal velocity values can be obtained through GPS and IMU information fusion, and errors generated by the IMU’s long integration time can be corrected, and real-time vehicle pose can be calculated by combining the track calculation method.

### 2.1. Yaw Angle and Longitudinal Velocity Estimation

This section focuses on estimation of the vehicle trajectory using an IMU and a GPS receiver. The vehicle velocity and yaw angle can be estimated by a sensor fusion algorithm using the data obtained from an IMU and a GPS. The main source of inertial sensor error is drift caused by sensor deviation and gravity effects. Therefore, the method in this paper aims to model these error sources and ignore the influence of cross-coupling errors and sensor scale factor errors. The IMU offers six degrees of freedom and consists of a three-axis gyroscope and a three-axis accelerometer which are installed on the carrier. In this paper, only the *z*-axis of the gyro and *x*-axis of the accelerometer are modeled as required. 

#### 2.1.1. Gyro Modeling

The output of the gyroscope can be expressed as the real vehicle yaw rate, with zero deviation and white noise, as shown in Equation (1):

(1) $$g_{r}=r+b_{r}+\omega_{gyro}$$

where, $g_{r}$ is the output of the gyro, r is the yaw rate of vehicle, $b_{r}$ is the constant offset or bias of the gyro, $\omega_{gyro}$ is the zero mean white noise of sensor. Assuming that the sensor noise obeys normally distributed, and the sampled covariance is $E\left[\omega_{gyro}^{2}\right]=\sigma_{gyro}^{2}$.

The deviation of the gyroscope is represented by a first order Markov process:

(2) $${\dot{b}}_{r}=-\frac{1}{T_{g}}\cdot b_{r}+\omega_{g\_bias}$$

where, $T_{g}$ is the correlation time. $\omega_{g\_bias}$ is the process driving noise of the gyro which is normally distributed with zero mean and a sampled covariance of $E\left[\omega_{g\_bias}^{2}\right]=\sigma_{b_{g}}^{2}$.

#### 2.1.2. Accelerometer Modeling

The accelerometer is modeled in the same way as the gyro. The influence of Coriolis acceleration and gravity acceleration were not considered in the modeling process:

(3) $$a=\ddot{x}+b_{a}+\omega_{accel}$$

where, a is the output of accelerometer, $b_{a}$ is the constant offset or bias of the accelerometer. $\omega_{accel}$ is the process driving noise of the accelerometer which is obeying normally distributed and the sampled covariance is $E\left[\omega_{accel}^{2}\right]=\sigma_{accel}^{2}$.

The accelerometer bias is also represented by a first order Markov process:

(4) $${\dot{b}}_{a}=-\frac{1}{T_{a}}\cdot b_{a}+\omega_{a\_bias}$$

where, $T_{a}$ is the correlation time. $\omega_{a\_bias}$ is the process driving noise of the accelerometer which is obeying normally distributed and the sampled covariance is $E\left[\omega_{a\_bias}^{2}\right]=\sigma_{b_{a}}^{2}$.

#### 2.1.3. Kalman Filter Establishment

Velocity, gyro bias, yaw angle and accelerometer zero bias were selected as state variables which are presented as $x={\left[\begin{array}{cccc} \psi & b_{r} & v & b_{a} \end{array}\right]}^{T}$. The longitudinal acceleration and yaw rate are the measurements of IMU, expressed as $u={\left[\begin{array}{cc} g_{r} & a \end{array}\right]}^{T}$. According to Equations (1) and (4), the equation of state of the system is:

(5) $$\dot{x}=Ax+Bu+\omega$$

where:

(6) A=[0−1000−1Tg00000−1000−1Ta]

(7) $$B={\left[\begin{array}{cccc} \begin{array}{c} 1\\ 0 \end{array} & \begin{array}{c} 0\\ 0 \end{array} & \begin{array}{c} 0\\ 1 \end{array} & \begin{array}{c} 0\\ 0 \end{array} \end{array}\right]}^{T}$$

The velocity and yaw angle measured by GPS are selected as external observation parameters and the system measurement equation is established as follows:

(8) y=Cx+μ

where, μ is the sensor noise, represented as $\mu ={\left[\begin{array}{cc} \mu_{\psi } & \mu_{v} \end{array}\right]}^{T}$ and it is satisfied that $E\left[\mu_{\psi }^{2}\right]=\sigma_{\psi }^{2}$ and $E\left[\mu_{v}^{2}\right]=\sigma_{v}^{2}$, respectively, where:

(9) $$y=\left[\begin{array}{c} \psi_{GPS}\\ v_{GPS} \end{array}\right]$$

(10) $$C=\left[\begin{array}{cccc} \begin{array}{c} 1\\ 0 \end{array} & \begin{array}{c} 0\\ 0 \end{array} & \begin{array}{c} 0\\ 1 \end{array} & \begin{array}{c} 0\\ 0 \end{array} \end{array}\right]$$

The covariance matrices Q and R of the process noise and the measured noise are solved, and the linear Kalman filter is used for the optimal estimation. Readers may refer to [41] for details. 

### 2.2. Vehicle Kinematics

The sensor fusion information is used to build the vehicle kinematics model, so as to obtain the vehicle trajectory. Firstly, the vehicle motion is simplified and described as a motion in a two-dimensional plane, as shown in Figure 1. The kinematics model uses three parameters to describe the motion of the vehicle, which represents the current abscissa X(t) of the vehicle, the current ordinate Y(t) of the vehicle and the vehicle’s current yaw angle ψ(t). The global coordinate system and the local coordinate system are respectively established at the center of mass of the vehicle. The horizontal axis of the global coordinate system is X and the vertical axis is Y. The horizontal axis of the local coordinate system is x and the vertical axis is y. In Figure 1, $x_{0}$ and $y_{0}$ are the local coordinate systems established by the vehicle at time $t_{0}$. ψ is the angle between the longitudinal axis of the vehicle and the X-axis. V is the velocity at the center of mass of the vehicle. $V_{X}$ and $V_{Y}$ are the projection of the vehicle velocity on the X-axis and Y-axis in the global coordinate system. The kinematics equation of the vehicle in the global coordinate system is:

(11) $$\dot{X}\left(t\right)=V\cos\left(\psi \left(t\right)-\beta \right)$$

(12) $$\dot{Y}\left(t\right)=V\sin\left(\psi \left(t\right)-\beta \right)$$

(13) $$\dot{\psi }\left(t\right)=\gamma$$

From Equations (11)–(13), it can be seen that the vehicle’s motion position is determined by the yaw rate, longitudinal acceleration of the center of mass and sideslip angle. 

In the global coordinate system, the vehicle position is described as $\left[\begin{array}{ccc} X & Y & \psi \end{array}\right]$. Assuming that the vehicle’s position at initial time $t_{0}$ is $P\left(t_{0}\right)={\left[\begin{array}{ccc} X\left(t_{0}\right) & Y\left(t_{0}\right) & \psi \left(t_{0}\right) \end{array}\right]}^{T}$, then the vehicle’s position at time $t_{1}$ can be expressed as follows:

(14) $$P\left(t_{1}\right)=\left[\begin{array}{c} X\left(t_{1}\right)\\ Y\left(t_{1}\right)\\ \psi \left(t_{1}\right) \end{array}\right]=\left[\begin{array}{c} X\left(t_{0}\right)+\int_{t0}^{t1}V_{X}\left(\tau \right)d\tau \\ Y\left(t_{0}\right)+\int_{t0}^{t1}V_{Y}\left(\tau \right)d\tau \\ \psi \left(t_{0}\right)+\int_{t0}^{t1}\gamma \left(\tau \right)d\tau \end{array}\right]$$

### 2.3. Vehicle Trajectory and Lane Polynomial

The vision sensor performs lane detection in a local coordinate system. Therefore, the vehicle trajectory and lane are defined in the local coordinate system of the vehicle. Lane curves and vehicle motion trajectories are shown in Figure 2.

Assuming that the vehicle is moving at constant velocity $V_{x}$ and yaw rate $\dot{\psi }$, the vehicle trajectory can be approximated by a parabolic projection. The vehicle trajectory $f_{v}\left(x\right)$ is expressed as follows:

(15) $$f_{v}\left(x\right)=\frac{\rho_{v}}{2}\cdot x^{2}=\frac{\dot{\psi }}{2\cdot V_{x}}\cdot x^{2}$$

At present, the general method is to describe the two-dimensional geometry of the lane through the cyclotron lines model. Taking an expressway as an example, the radius of lanes is generally more than 100 m, so the curvature and curvature rate are usually small and the geometry of the lane can be expressed by a cubic polynomial equation. Through the cubic polynomial, the left and right lanes can be described as follows:

(16) $$f_{L}\left(x\right)=c_{L0}+c_{L1}\cdot x+c_{L2}\cdot x^{2}+c_{L3}\cdot x^{3}$$

(17) $$f_{R}\left(x\right)=c_{R0}+c_{R1}\cdot x+c_{R2}\cdot x^{2}+c_{R3}\cdot x^{3}$$

where, $c_{L0}$ and $c_{R0}$ represent the lateral offset between the vehicle and the left lane or right lane at the current moment, respectively. The terms $c_{L1}$ and $c_{R1}$ represent the heading angle between the vehicle and the left lane or right lane at the current moment, respectively, while $c_{L2}$ and $c_{R2}$ represent the curvature of the left lane or right lane at the current moment, respectively and $c_{L3}$ and $c_{R3}$ represent the curvature rate of the left lane or right lane at the current moment, respectively. 

Taking the average value of the left and right lanes and then the polynomial of the road centerline $f_{M}\left(x\right)$ is shown as follows:

(18) $$f_{M}\left(x\right)=c_{0}+c_{1}\cdot x+c_{2}\cdot x^{2}+c_{3}\cdot x^{3}$$

where, $c_{0}=\left(c_{L0}+c_{R0}\right)/2$; $c_{1}=\left(c_{L1}+c_{R1}\right)/2$; $c_{2}=\left(c_{L2}+c_{R2}\right)/2$; $c_{3}=\left(c_{L3}+c_{R3}\right)/2$.

## 3. Lane Parameters Estimation

The system is a multi-rate system. The visual sensor, IMU, GPS and vehicle controller operate at different update rates, and the data can be obtained through the vehicle CAN bus. The information transmission of sensors and controllers is shown in Figure 3.

In Figure 3, the update rate of vision sensor is $T_{cam}$, the update rate of IMU is $T_{c}$, and the update rate of GPS is $T_{G}$. The relationship between the three update rate is $T_{G}>T_{cam}>T_{c}$. Since the Kalman filter and IMU operate at the same rate, we only focus on the relationship between $T_{cam}$ and $T_{c}$. Assuming that there is an integer n(n>1) that makes $T_{cam}=n\cdot T_{c}$, according to the difference of update rate between IMU and the camera sensor which shown in Figure 4, the time constant t is defined as:

(19) $$t=\left(k+\frac{i}{n}\right)T_{cam}$$

where, k(k=0,1,⋯) and i(i=0,1,⋯n−1) represent the update periods of the vision sensor and IMU, respectively.

It is assumed that the vision sensor at time k can obtain stable lane information, and the longitudinal velocity and yaw angle can be obtained after the fusion of IMU and GPS data. Based on the difference in the sensor update rate, the vehicle trajectory can be continuously calculated within the interval of the vision sensor update. Assuming that the initial vehicle position at time k is $P\left(t_{0}\right)={\left[\begin{array}{ccc} 0 & 0 & 0 \end{array}\right]}^{T}$, the equation of vehicle position at time k+1 can be expressed as follows after discrete processing:

(20) $$\hat{\psi }\left(k|i\right)=\sum_{j=0}^{i}\psi \left(k|j\right)$$

(21) $$\hat{x}\left(k+1|0\right)=\sum_{i=0}^{n-1}V_{x}\left(k|i\right)\cdot \cos\left(\hat{\psi }\left(k|i\right)\right)\cdot T_{c}$$

(22) $$\hat{y}\left(k+1|0\right)=\sum_{i=0}^{n-1}V_{x}\left(k|i\right)\cdot \sin\left(\hat{\psi }\left(k|i\right)\right)\cdot T_{c}$$

where $V_{x}$ is the component of the speed V in the local coordinate system of the vehicle.

Vehicle position and trajectory equation are solved by using Equations (15) and (20)–(22). The prediction method is derived below to predict the coefficient of lane polynomial at time k+1. 

### 3.1. Lateral Offset Estimation

In the local coordinate system, the relationship between the vehicle center of mass and the lane is used to predict the lane coefficient, which is shown in Figure 5.

The vertical line of the tangent line of the vehicle trajectory at point $P_{k+1}$ intersects the lane at point $Q_{k+1}$. g(x) is the line passing through the point $P_{k+1}$ and point $Q_{k+1}$:

(23) g(x)=ax+b

In the plane rectangular coordinate system, the angle between g(x) and the *x*-axis is $\frac{\pi }{2}+\hat{\psi }\left(k+1\right)$, and the slope and intercept are expressed as *m* and *b*, respectively:

(24) $$a=\tan\left(\frac{\pi }{2}+\hat{\psi }\left(k+1|0\right)\right)$$

(25) $$b=\hat{y}\left(k+1|0\right)-m\cdot \hat{x}\left(k+1|0\right)$$

For simultaneous Equations (18) and (23):

(26) $$c_{0}+c_{1}\cdot x+c_{2}\cdot x^{2}+c_{3}\cdot x^{3}=ax+b$$

The horizontal coordinate of point $Q_{k+1}$ can be solved that using the secant method. Let’s define the coordinates $Q_{k+1}\left({\hat{x}}_{Q}\left(k+1|0\right),f_{L}\left({\hat{x}}_{Q}\left(k+1|0\right)\right)\right)$. Then, the Euclidean distance between $P_{k+1}$ and $Q_{k+1}$ can be obtained, namely, the lateral offset ${\hat{c}}_{0}\left(k+1|0\right)$:

(27) $${\hat{c}}_{0}\left(k+1|0\right)=\mathrm{sgn}\left(f_{L}\left({\hat{x}}_{Q}\left(k+1|0\right)\right)\right)\cdot \sqrt{X_{e}{}^{2}+Y_{e}{}^{2}}$$

where:

(28) $$X_{e}={\hat{x}}_{Q}\left(k+1|0\right)-\hat{x}\left(k+1|0\right)$$

(29) $$Y_{e}=f_{L}\left({\hat{x}}_{Q}\left(k+1|0\right)\right)-f_{v}\left(\hat{x}\left(k+1|0\right)\right)$$

### 3.2. Heading Angle Estimation

As shown in Figure 5, the heading angle is the angle between the tangent line of the vehicle trajectory and the tangent line of the lane. Using geometric relations, the heading angle ${\hat{c}}_{1}$ is calculated by solving the slope of the tangent line at the points $P_{k+1}$ and $Q_{k+1}$:

(30) $$\tan\left(\theta_{1}\left(k+1|0\right)\right)=f_{v}^{\prime }\left(x\right){|}_{x=\hat{x}\left(k+1|0\right)}$$

(31) $$\tan\left(\theta_{2}\left(k+1|0\right)\right)=f_{L}^{\prime }\left(x\right){|}_{x={\hat{x}}_{Q}\left(k+1|0\right)}$$

As shown in Figure 5, ${\hat{c}}_{1}\left(k+1,0\right)$ is the error between $\theta_{1}\left(k+1,0\right)$ and $\theta_{2}\left(k+1,0\right)$, and the tangent value of the angle is presented as follows,

(32) $$\tan\left({\hat{c}}_{1}\left(k+1|0\right)\right)=\tan\left(\theta_{1}\left(k+1|0\right)-\theta_{2}\left(k+1|0\right)\right)=\frac{m_{1}-m_{2}}{1+m_{1}m_{2}}$$

where, *m*_1_ = tan(*θ*_1_(*k* + 1|0)), *m*_2_ = tan(*θ*_2_(*k* + 1|0)).

When the heading angle is small, ${\hat{c}}_{1}\left(k+1|0\right)$ can be approximately equal to:

(33) $${\hat{c}}_{1}\left(k+1|0\right)=\tan^{-1}\left(\frac{m_{1}-m_{2}}{1+m_{1}m_{2}}\right)\approx \frac{m_{1}-m_{2}}{1+m_{1}m_{2}}$$

### 3.3. Curvature and Curvature Rate Estimation

According to the design characteristics of expressway, it is approximately considered that the curvature rate of lane is constant in a single period. According to Equation (18), $f_{L}^{\prime \prime }\left(x\right)=2c_{2}+6c_{3}\cdot x$, the vehicle position at the current moment is zero in the local coordinate system of the vehicle, so $f_{L}^{\prime \prime }\left(0\right)=2c_{2}$. Then we will calculate the curvature and curvature rate at time k+1:

(34) $${\hat{c}}_{2}\left(k+1|0\right)={\ddot{f}}_{L}\left(x\right){|}_{x=\hat{x}\left(k+1|0\right)}=2c_{2}\left(k|0\right)+6c_{3}\left(k|0\right)\hat{x}\left(k+1|0\right)$$

(35) $${\hat{c}}_{3}\left(k+1|0\right)=\frac{{\hat{c}}_{2}\left(k+1|0\right)-c_{2}\left(k|0\right)}{\kappa }$$

where, κ is an tuning parameter related to vehicle speed, and the value is approximately equal to the sampling time of the vision sensor. 

If the sensor fails to provide lane information within several sampling cycles, the predictive compensation method derived above is used for road compensation. However, when the sensor is ineffective for a long time, the performance of lane prediction will decline due to the lack of road information feedback.

## 4. Experimental Results

The method is evaluated by hardware-in-the-loop simulation platform and vehicle experiments.

### 4.1. Simulation

In the hardware-in-the-loop simulation, Carsim software is used to simulate a A-class vehicle. In the simulation process, the velocity is set to 25 m/s (i.e., 90 km/h). The expected path is a third-order polynomial curve that conforms to cyclotron constraints. The parameters used in Carsim are the nominal values of the test vehicle. The HIL platform is shown in Figure 6, and the HIL process is shown in Figure 7. 

As shown in Figure 7, the 27-DOF nonlinear vehicle model of Carsim is used to simulate the virtual vehicle. The state input of vehicle, feedback of steering controller and compensation algorithm all run in AutoBox which from dSPACE. The communication between each part is realized by using CAN bus.

The prediction performance of the method is verified based on the HIL platform, and the vehicle steering change process caused by sensor failure during lane restore is simulated. In the process of simulation, the following three scenarios were considered: (a) The vision sensor can detect the road information normally; (b) the vision sensor fails every 10 s, and the failure time is variable; (c) when the vision sensor fails, the compensation algorithm is used to restore the lane. 

Figure 8 shows the comparison of lateral offset, heading angle, curvature and curvature rate in the three scenarios. The blue line shows the data measured by the virtual sensor. The red line shows the measured data which contains the failure of the virtual sensor. The green line shows the data predicted using the compensation algorithm. On the road, the failure occurred at 5, 15, 25, 35, 45 and 55 s, respectively. The first 50 s shown in the figure are a variable curvature road and the remaining time is an approximately straight road. The results show that the method can achieve good results on both straight and curved roads.

Figure 9 shows the errors between the measured data and the restored data. On the road, the failure occurred in 5, 15, 25, 35, 45 and 55 s, respectively. The first 50 s shown in the figure are variable curvature road and the remaining time is an approximately straight road. The results show that the method can achieve good results on straight and curved roads. The statistical information of the errors is shown in Table 1. The lateral displacement of the error is less than ±2 × 10^−2^ m, heading angle error is less than ±4 × 10^−4^ rad, curvature of the error is less than ±1.2 × 10^−5^ m^−1^, the error of the curvature change rate is less than 1.5 × 10^−7^ m^−2^. The RMSE of each variable is far less than the magnitude of the error. This indicates that the predicted lane is very close to the compensated lane. The steering angle error caused by the maximum prediction error is far less than 1°, so the influence of the prediction error on the control accuracy can be neglected.

Considering the safety, HIL is used to verify the lane-keeping based on compensation method. We design a lane keeping controller based on PID theory. In the program, bad points are set manually. In Figure 10, the blue line indicates lane-keeping control with sudden bad points, while the red dotted line represents lane-keeping control after compensation by the algorithm and the tracking effect is represented by steering wheel angle. At 25 s, due to the appearance of bad points, the uncompensated control produces the sudden change of steering wheel angle, which leads to the instability of the controlled vehicle and easily causes accidents. After compensation, the control effect is stable, and the vehicle smoothly transits to the sensor and returns to normal. 

### 4.2. Vehicle Test

Figure 11 shows the experimental vehicle and the experimental road section. The experimental vehicle is equipped with sensors such as Mobileye, IMU and GPS. The update rate of each sensor is shown in Table 2. The update periods of ECU controller, visual sensor, IMU and GPS are all different. This is a typical multi-rate system. The ECU controller communicates with the sensors through the CAN bus. The vehicle velocity is controlled between 60 km/h and 70 km/h. The prediction method is compared with the measured data of the vision sensor. The characteristics of the experimental road are as follows:

- Total length: 4000 m (straight line section: 1500 m; curve line section: 2500 m)
- Width: 2- lane (each lane width is 3.5 m)
- Curve radius: 250 m and 400 m.

Figure 12 shows the performance of the estimation method in a vehicle test. The red line shows the measured data by the vision sensor. The blue dots line shows the estimated data by the compensation algorithm. In the test process, when one of the two lines cannot be detected, it is also considered a failure. It can be seen that the compensation effect is good in straight and curve sections.

Figure 13 shows the lane estimation between 20 s to 30 s in four frames. The blue lines represent the lane measured by the camera. The black dot lines represent the center lane which calculated by the left and right line. The green asterisk indicates that when the camera fails temporarily, the method proposed in this paper can better predict the lane. The predicted lane meets the requirements of lane keeping control.

## 5. Conclusions

In this study, a lane compensation method based on sensor fusion is proposed to compensate for the short-time failure of vision sensors. The method is divided into two parts. The first part is the vehicle trajectory acquisition based on sensor fusion, and the second part is the lane prediction using the relative position of the vehicle and road. The hardware-in-the-loop and vehicle experiments show that the short-time failure of vision sensors can be compensated by this method.

The algorithm has two main contributions. Firstly, a lane compensation method based on sensor fusion is proposed. That is, through the fusion of low-cost sensors, high-precision vehicle status information can be obtained, and then the relative position of vehicles and roads can be used to predict the road coefficient. Secondly, the simulation and vehicle experiments are used to verify the effectiveness and real-time performance of the lane compensation algorithm. It validates the applicability of the algorithm in the case of discontinuous bad points and short duration of bad points.

In the future, we will use more complex working conditions to verify the algorithm and consider combining other sensors to extend the compensation time. Based on this, we will consider the impact of speed on the algorithm to improve the compensation method. In addition, lane detection method will also be focus of our research.

## Figures and Tables

**Figure 1:** Vehicle kinematics model.

**Figure 2:** Vehicle trajceotry and lane polynomial.

**Figure 3:** System block diagram.

**Figure 4:** Update periods of the IMU and camera sensor.

**Figure 5:** Relationship between vehicle’s trajectory and lane polynomial.

**Figure 6:** HIL platform.

**Figure 7:** Flow chart of HIL.

**Figure 8:** Contrast in three scenarios

**Figure 9:** Errors between measured and restored values.

**Figure 10:** Comparison of steering wheel angle.

**Figure 11:** Experimental vehicles and test sites.

**Figure 12:** Lane test results.

**Figure 13:** Lane estimation at time k, k + 2, k + 4, k + 6.

**Table 1:** Lane prediction results.

	Error Boundaries	RMSE
Lateral offset [m]	1 × 10^−2^	3.9 × 10^−3^
Heading angle [rad]	4 × 10^−4^	1.18 × 10^−4^
Curvature [1/m]	1.2 × 10^−^^5^	4 × 10^−^^6^
Curvature rate [1/m^2^]	1.5 × 10^−^^7^	3.24 × 10^−^^8^

**Table 2:** Update period of sensor.

Sensor/Parameters	Update Period (ms)
ECU	10
Vision (Mobileye)	70
GPS (Trimble)	500
IMU (BOSCH)	10
